This article has been retracted.

# An AI-Enabled Internet of Things Based Autism Care System for Improving Cognitive Ability of Children with Autism Spectrum Disorders

**DOI:** 10.1155/2022/2247675

**Published:** 2022-05-23

**Authors:** Mohamed Abdel Hameed, M. Hassaballah, Mosa E. Hosney, Abdullah Alqahtani

**Affiliations:** ^1^Department of Computer Science, Faculty of Computers and Information, Luxor University, Luxor, Egypt; ^2^Department of Computer Science, Faculty of Computers and Information, South Valley University, Qena, Egypt; ^3^Department of Computer Science, College of Information Technology, Misr University for Science & Technology, Giza, Egypt; ^4^Department of Information System, Faculty of Computers and Information, Luxor University, Luxor, Egypt; ^5^College of Computer Engineering and Sciences, Prince Sattam Bin Abdulaziz University, Alkhrj, Saudi Arabia

## Abstract

Smart monitoring and assisted living systems for cognitive health assessment play a central role in assessment of individuals' health conditions. Autistic children suffer from some difficulties including social skills, repetitive behaviors, speech and nonverbal communication, and accommodating to the environment around them. Thus, dealing with autistic children is a serious public health problem as it is hard to determine what they feel with a lack of emotional cognitive ability. Currently, no medical treatments have been shown to cure autistic children, with most of the social assistive research to date focusing on Autism Spectrum Disorder (ASD) without suggesting a real treatment. In this paper, we focus on improving cognitive ability and daily living skills and maximizing the ability of the autistic child to function and participate positively in the community. Through utilizing intelligent systems based Artificial Intelligence (AI) and Internet of Things (IoT) technologies, we facilitate the process of adaptation to the world around the autistic children. To this end, we propose an AI-enabled IoT system embodied in a sensor for measuring the heart rate to predict the state of the child and then sending the state to the guardian with feeling and expected behavior of the child via a mobile application. Further, the system can provide a new virtual environment to help the child to be capable of improving eye contact with other people. This way is represented in pictures of these persons in 3D models that break this child's fear barrier. The system follows strategies that have focused on social communication skill development particularly at young ages to be more interactive with others.

## 1. Introduction

Cognitive impairment is a brain condition resulting from trauma such as old age, falls, road accidents or sports-related injuries, or other causes, including vascular, infective, or inflammatory insults [1]. Some signs of cognitive impairment are memory concerns, or other cognitive complaints. Cognitive assessment assists individuals who cannot efficiently carry out their routine activities to promote sustainability and support independent living. Nowadays, intelligent systems based AI technologies are widely used in smart cognitive health and medical applications for health monitoring of individuals with diseases to avoid possible risks [2]. These AI based systems do not complain fatigue; thus, they can process large quantities of data at very high speed outperforming humans accuracy in the same job [3, 4]. Machine learning and AI techniques are used in medical technologies to improve the diagnostic capability of clinicians, especially in multidisease diagnosis [5–9]. With progress in employing intelligent AI systems with help of IoT in healthcare, patients can be diagnosed professionally and faster; thus, they may start treatment sooner. On the other hand, IoT has been the key part of the Internet [10, 11]. It has been used in many domains such as identifying objects, determining the location and sensing changes in physical data. The descriptive models for IoT are introduced based on two attributes (“being an Internet”, “relating to thing's information”) and different features based on the thing's information [12, 13].

Autism is a neurological disorder that affects the ability to communicate and interact socially. It can be defined as a neurobehavioral condition that involves weaknesses in communication skills and social interaction and developmental language combined with repetitive behaviors. Because of the range of symptoms, this is called Autism Spectrum Disorder (ASD) [14, 15]. The cause of the increasing number of autistic children is not yet known. However, early intervention is critical to enabling a positive long-term outcome, and even with early intervention, many individuals will need high levels of support and care throughout their lives [16, 17]. Children with difficulties in relating and communicating may fall within a wide series of disorders such as autistic spectrum disorder, language processing disorders, attention disorders, and sensory or regulatory disorders. The child gets a diagnosis established by the observation of the behaviors outlined above. Although the child may share a common diagnosis with others, each child is unique in his processing of sensory as a unique pattern of development and functioning [18, 19].

One of the difficulties we face when dealing with the children is to determine what they feel, especially autistic children, as those with this disease suffer from a difficulty in accommodating to the environment around them. One way to overcome this problem is by using assistive technologies and finding ways how to benefit from the use of technology of intelligent systems to help these children. An assistive smart environment has the effort to improve the quality of life for large populations of users: elderly, individuals with physical impairments, and individuals with cognitive disabilities and developmental and social disorders [20, 21].

The primary goal of this research is to establish a supportive environment using IoT and AI technology to help autistic children in communicating with others in an easy and flexible way. The main problem of autistic children is considered in expressing their feelings and in communicating with others. Also, they suffer from an inability to connect visually. Thus, we suggest a new technical solution to help them interact with people visually and use the technology to make this easy for interaction. It can be done by using computer graphics to make a three-dimensional model that simulates the real person, whom we want the autistic child to interact with visually and acoustically.

In this paper, we proposed and implemented an intelligent system prototype based on machine learning algorithms and an assistive smart environment for promoting learning and developing interaction with autistic children life. The main objective is to convert the child's state to emotion and send it to the guardian. Looking for the best way to know the state of the person, we found that the heart rate reading is the most accurate. So, we choose sensor “Heartbeat” for reading the heart rate because it is easy, accurate, and practical in use. This sensor is embodied in the form of a hand watch to be suitable for children, and it will read the heart rate, which is converted to numeric values representing the heart rate. These values are classified by the retrained classification models. Then, based on the classification result, a message is sent with the state of child feeling via mobile application to the guardian or a charge person. Also, the system will help in affording different activities of the child with scheduling and alerting the mother when it is time. Further, the system can provide a new virtual environment to help the child to be capable of improving eye contact with other people. This way is represented in pictures of these persons in 3D models that break the child's fear barrier. The system follows strategies that have focused on social communication skill development particularly at young ages from 4 to 12 years to be more interactive with others.

The rest of the paper is organized as follows: Section 2 discusses the related works.  Section 3 gives details of the materials and methods used in the proposed system.  Section 4 explains the main modules containing hardware and software implementation of the proposed system. In Section 5, the experimental results and discussion are presented. Finally, the paper is concluded in Section 6.

## 2. Related Work

The first study in ASD therapy or diagnosing diseases was published around the 1960*s* when autism was thought to be a very dangerous condition resulting from intellectual disability [22]. These studies reported the spread to be approximately four to five cases per 10,000 children. In [23], autism was identified as a novel clinical diagnosis by the American Psychiatric Association, which provided pervasive developmental disorder and diagnostic principles for childish autism.

Rasche and Qian [24] identified and distinguished the territories of mental imbalance in the areas of autism therapy that can be upgraded and improve the learning background of the autistic children. The technology involved in this proposed project is a Touch Screen Mobile Computer (TSMC) device, which plays a critical role in enhancing the autistic child's learning experience. The idea is to use TSMC as an instructional tool to explore the viable implementation and improvise the learning experience of children with ASD at inexpensive price.

In [25], the authors present the design and implementation of a smart device called “Things that think” (T3), which converts traditional objects into smart objects that promote interactivity with playful and engaging interaction. Smart objects can help teachers overcome the problems encountered during the object recognition training of students with autism disorder. The idea in [26] is designed to save women or children in hazard by alerting in the mode of notification, which is sent through a wearable device. This system involves the technology GSM or GPS module for location tracking purposes and various sensors such as pulse rate sensor, temperature sensor, and motion sensor for monitoring the heartbeat and detecting the pulse condition of the person.

Shi et al. [27] proposed a system for enhancing the interactions among children with ASD and overcome the lack of interaction between the autistic children. The main goal of the work is to provide services on data-driven detection, therapy, intervention, and monitoring the ASD children. The purpose of detecting the interaction between the autistic children provided the sensor framework comprises of sensor badges worn by child and teacher participants in the pockets of the customized T-shirt. In [28], the authors proposed an assistive involvement for supporting the overloaded sensory responses in individuals with ASD, namely, Assistive Companion for Hypersensitive Individuals (ACHI). Also, the ACHI technology can help the autistic children to become calm.

Popescu et al. [29] proposed machine learning-based mobile application called PandaSays, which was improved and integrated with an Alpha 1 Pro robot, and discussed the performance evaluation using deep convolutional neural networks and residual neural networks. The model trained with MobileNet convolutional neural network had an accuracy of 56.25%, performing better than ResNet50 and VGG16. In [30], an important technique for analyzing machine learning algorithms was used, in order to predict Autism Spectral Disorder (ASD) disease in a competent yet convenient way. Discriminant analysis algorithms are investigated, and well-organized analytical models are fabricated with LDA and QDA with hyperparameter tuning for better upshots. The accuracy of QDA is 71.82%, which, after tuning, bolsters the maximum accuracy of 99.77% leaving behind LDA in terms of other performance metrics too.

More recently, Farhan et al. [31] illustrated how the use of the NAO robots improves the verbal and nonverbal communication of children with autism. In this research, four children from Welfare of Autistic Children (SWAC, Dhaka, Bangladesh) participated, and four sessions were held. The first session was referred to the introduction of the robot, and the second session had the purpose of getting answers from the children. The NAO robot asked the children some of the following questions: “How old are you?” “How are you?” “What is your father's name?” “What is your name?” And “What is your mother's name?” The third session was dedicated to physical activities, such as dancing and exercising, and the fourth session was about gathering feedback regarding sessions 2 and 3. After four weeks, the overall performance increased by 45% in the first child, 70% in the second child, 30% in the third child, and 75% in the fourth child.

## 3. Materials and Methods

This section presents materials and methods used to implement the proposed system including hardware components, feature extraction and selection, IoT, and classification based machine learning algorithms.

### 3.1. Hardware Requirements

The hardware shown in Figure 1 that has been used to build the proposed system is as follows:

1. Arduino Uno R3 (ESP32).
2. Heartbeat sensor.
3. Breadboard and jumper wires.

#### 3.1.1. Arduino Uno R3 (ESP32)

The Arduino Uno *R*3 model ESP32 shown in Figure 1 is used, where R3 is the third revision of the Arduino. ESP32 [32] provides the following key features:

1. Ultra-Low Power Consumption: ultra-low power of ESP32 is achieved according to the combination of several types of proprietary software. It is designed for mobile devices, wearable electronics, and IoT applications.
2. Robust Design: it can function reliably in industrial environments, with an operating temperature ranging from −−40*C* to +125*C*.
3. High Level of Integration: it is highly integrated with built-in antenna switches, power amplifier with low-noise receiver, and power management modules.
4. Hybrid Wi-Fi and Bluetooth Chip: it can perform as a complete standalone system or as a slave device to a host multipoint control unit, reducing communication stack overhead on the main application processor.

#### 3.1.2. Heartbeat Sensor

A heartbeat sensor is an electronic device used to measure the speed in beat per minute (BPM). Heartbeat is monitored in two ways: a manual way where the heartbeat can be exploited by checking one's pulses at two locations, wrist and the neck; the other way where the heartbeat can be measured by using a sensor that is based on optical power variation as light is scattered or absorbed during its path through the blood as the heartbeat changes [33, 34]. The pulse sensor is used to collect heart rate data and pulses from the human body. This sensor includes the *LED*, which blinks according to the pulses that contain some noise. This noise is discarded using *noise elimination circuitry* [35].

### 3.2. Internet of Things

IoT is usually represented as a key part of the future Internet and radio frequency identification (RFID) tags and is used to identify objects uniquely, for determining the location and sensing changes in physical data, which is used later for communicating with the intended receiver [28]. The interactions with autistic children are considered as one of the most difficult and challenging problems which their families and caregivers deal with. IoT is introduced as an emerging technology for the modern information age. In health-care, some wearable sensors are used for many purposes not only for monitoring the body parameters like heart rate, but also for storing the obtained data for decision-making. The main components for this technology are cloud computing, IoT, and Wireless Body Area Network (WBAN). Children with ASD like Alzheimer's patients and dementia suffer from forgetfulness, so they tend to get into dangerous situations as escaping from home. Children with ASD could avoid leaving their safe zone by using this technology, so they proposed the Alzimio application for solving these kinds of problems utilizing IoT devices. Data mining methods such as classification, regression, and clustering for early detection of ASD are applied so early diagnosis of ASD, which becomes an important factor for providing appropriate education and also support services to patients and their caregivers [36].

### 3.3. Feature Extraction

Feature extraction offers a set of features from a high-dimensional space into a shortened set of features from a low-dimensional space, while the data is still describing with adequate accuracy. Furthermore, feature selection algorithms could be linear or nonlinear [37]. Linear methods perform mapping of the linear data to a lower-dimensional space such as Principal Component Analysis (PCA) and Linear Discriminant Analysis (LDA) [38]. PCA increases the original information of the data after dimension reduction and decides the importance of this direction by measuring the variance of the data in the projection direction. However, such projections may not be good enough to differentiate classes of data. Instead, they may make data points blend together and be the same. PCA essentially finds better projection methods from the perspective of the covariance of features [39] and can be calculated as follows:

Calculate the mean *μ* and standard deviation *σ* of feature as

(1) $$\begin{array}{c} x_{\text{new}}=\frac{x-\mu }{\sigma }. \end{array}$$

Calculate the covariance matrix Cov(*x*, *y*) for the features in the dataset by using

(2) $$\begin{array}{c} \text{Cov}\left(x,y\right)=\frac{\sum \left(x_{i}-\bar{x}\right)*\left(y_{i}-\bar{y}\right)}{N}. \end{array}$$

Then, find the eigenvalues *λ* of the covariance matrix and arrange them in a descending order, *λ*_1_ ≥ *λ*_2_ ≥ ⋯≥*λ*_*d*_ with the corresponding eigenvectors {**A**_1_, **A**_2_,…, **A**_*d*_}.

Choose *k* eigenvectors with the largest eigenvalues *λ*, where *k* is the number of dimensions of the *x*_new_ dataset. Then, transform the original matrix using

(3) $$\begin{array}{c} \text{Final Data }=\text{ Feature matrix }*\text{ high }k\text{ eigenvectors.} \end{array}$$

### 3.4. Feature Selection

Any machine learning algorithm can perform classification by using a set of features. This feature is known as a singular measurable property of the process being observed [40]. Mainly, feature selection is used as a process for decreasing the number of input variables during improving a predictive model. It uses variable ranking methods for selection according to an ordering scheme. Moreover, ranking methods are applied before classification to filter out the less related variables, reducing the computational cost of modeling and developing the efficiency of the model. To achieve this, a subset of variables is selected from the input, which can efficiently define the input data while decreasing effects from noise or unnecessary variables and still providing good prediction results [41]. The feature selection methods are broadly classified into three categories according to user data sets as, filter, wrapper, and embedded selection methods, respectively.

Filter methods are run as preprocessing to list the features, wherein the highly ranked features are selected and applied to a predictor. The ranking measure is used to obtain the variables with a threshold value, which is used to remove variables less than it. This feature contains useful information about the different classes in the data, which lead to speed and ability to scale in the large datasets [40]. The formula of filtering normalization can be computed using the following steps:

**Step 1 .**

Identify the minimum and maximum value in the dataset *x*_min_ and *x*_max_, respectively.

**Step 2 .**

Calculate the range of the dataset by subtracting the minimum value from the maximum value as

(4) $$\begin{array}{c} \text{Range}=x_{\max}-x_{\min}. \end{array}$$

**Step 3 .**

Determine how much more values in the variable to be normalized from the minimum value *x* − *x*_min_.

**Step 4 .**

Finally, the normalized *x* is derived by dividing the expression in step 3 by the one in step 2 as

(5) $$\begin{array}{c} X_{\text{normalized }}=\frac{\left(x-x_{\text{min}}\right)}{\left(x_{\text{max}}-x_{\text{min}}\right)}. \end{array}$$

On the other hand, wrapper methods are the second type of the feature selection, where the predictor is wrapped on a search algorithm, which can find a subset that gives the highest predictor performance [42]. These methods are very useful with small training sets in which they may overfit. The last type of feature selection is the embedded methods, which contain variable selection as part of the training process without splitting the data into training and testing sets. So, it can be used to reduce the computation time taken up for reclassifying different subsets, which are done in wrapper method [40, 41]. In the proposed system, we use a filter method for feature selection to achieve low complexity and maintain the performance of the proposed system.

### 3.5. Machine Learning Algorithms

Machine learning and deep learning have been considered for classification tasks in several applications [43–45]. In this work, some machine learning classification algorithms, namely, random forest, K-nearest neighbors, and support vector machine, are utilized to determine the best classification model. The best classification algorithm should be able to achieve the better accuracy in classification for the given dataset, which can help classify the dataset for training and testing sets.

#### 3.5.1. Random Forest

The random forest algorithm is composed of different decision trees, each with the same nodes, but using different data that leads to different leaves. It merges the decisions of multiple decision trees in order to find an answer, which represents the average of all these decision trees. The random forest algorithm is a supervised learning model; it uses labeled data to “learn” how to classify unlabeled data. This is the opposite of the K-means cluster algorithm, which is an unsupervised learning model. In case of using the random forest algorithm to solve regression problems, the mean squared error can be used to split data branches into each node.

(6) $$\begin{array}{c} \text{MSE}=\frac{1}{N}\sum_{i=1}^{N}{\left(f_{i}-y_{i}\right)}^{2}, \end{array}$$

where *N* is data points, *f*_*i*_ is the value returned by the model, and *y*_*i*_ is the actual value for data point *i*.

For utilizing random forest for classification step, we use the Gini index to decide how to split nodes of a decision tree, where

(7) $$\begin{array}{c} \text{Gini}=1-\sum_{i=1}^{C}{\left(p_{i}\right)}^{2}. \end{array}$$

where *p*_*i*_ represents the relative frequency of the class, and *C* represents the number of classes.

On the other hand, the entropy can be used to determine number of nodes that branch in a decision tree by using

(8) $$\begin{array}{c} \text{Entropy}=\sum_{i=1}^{C}-p_{i}*\;\log_{2}\left(p_{i}\right). \end{array}$$

Entropy uses the probability of a certain outcome to make a decision on how the node should branch. Unlike the Gini index, it is more mathematical intensive due to the logarithmic function used in calculating it.

#### 3.5.2. K-Nearest Neighbors

This algorithm is one of the simpler techniques used in machine learning. It is preferred by many areas in the industry because of its ease of use and low calculation time. It is a model that classifies data points based on the points that are most similar to them. It uses test data to make an educated guess on what an unclassified point should be classified as. It is often used in simple recommendation systems, image recognition technology, and decision-making models. When implementing KNN, the data points are transformed into feature vectors or their mathematical value. Then, the algorithm works by finding the distance between the mathematical values of these points by using the Euclidean distance as

(9) $$\begin{array}{c} d\left(p,q\right)=d\left(q,p\right),\\ =\sqrt{{\left(q_{1}-p_{1}\right)}^{2}+{\left(q_{2}-p_{2}\right)}^{2}+\cdots +{\left(q_{n}-p_{n}\right)}^{2}},\\ =\sqrt{\sum_{i=1}^{n}{\left(q_{i}-p_{i}\right)}^{2}.} \end{array}$$

#### 3.5.3. Support Vector Machine

SVM is a supervised machine learning algorithm that showed high performance by many as it produces significant accuracy with less computation power, supporting vector machine. It can be used for both classification and regression challenges [46]. Besides, it is a maximum margin classifier, meaning that it increases the separation between *n* classes of data efficiently in a high-dimensional space in which the distinction between groups is nonlinear. So, the SVM algorithm is used in our model because of its direct geometric interpretation, being working very well with limited data set, and elegant mathematical tractability [47]. In general, SVMs have been shown to improve the accuracy of diagnoses classification. Also, they provide insight into how different characteristics can help distinguish between patients with and without ASD, for example, regulated assessments, eye movement data, neuroimaging data, upper limb, and general kinesthetic data. Currently, regulated assessments reliant on behavioral observation are the clinical standard for diagnosing ASD [48]. In the proposed system, we have used kernel SVM that contains a nonlinear transformation function to convert the complicated nonlinearly separable data into linearly separable data. In this context, a hyperplane in an n-D feature space [49] can be represented by

(10) $$\begin{array}{c} f\left(x\right)=x^{T}w+b=\sum_{i=1}^{n}x_{i}w_{i}+b=0. \end{array}$$

Dividing by ‖**w**‖, we get

(11) $$\begin{array}{c} \frac{x^{T}w}{\left\|w\right\|}=P_{w}\left(x\right)=-\frac{b}{\left\|w\right\|}. \end{array}$$

indicating that the projection of any point **x** on the plane onto the vector **w** is always −*b*/‖**w**‖, i.e., **w** is the normal direction of the plane, and |*b*|/‖**w**‖ is the distance from the origin to the plane. Note that the equation of the hyperplane is not unique. cf(**x**)=0 represents the same plane for any *c*. The *n*-D space is partitioned into two regions by the plane. Specifically, we define a mapping function *y*=sign(*f*(**x**)) ∈ {1, −1}, where

(12) $$\begin{array}{c} \begin{array}{c} f\left(x\right)=x^{T}w+b,\\ =\left\{\begin{array}{cc} >0, & y=\text{sign}\left(f\left(x\right)\right)=1,\;x\in P,\\ <0, & y=\text{sign}\left(f\left(x\right)\right)=-1,\;x\in N. \end{array}\right. \end{array} \end{array}$$

Any point **x** ∈ *P* on the positive side of the plane is mapped to 1, while any point **x** ∈ *N* on the negative side is mapped to −1. A point **x** of unknown class will be classified to *P* if *f*(**x**) > 0, or *N* if *f*(**x**) < 0.  Figure 2 shows the linear classification on two-dimensional dataset. There were many other variants of the SVM developed and widely used by the researchers for different issues such as binary SVM, multiclass SVM, and stacking SVM [49].

### 3.6. IBM Watson Assistant for Graphics Designer

The increasing number of children with an ASD is associated with some factors as parent distress and increased family chaos. The successful long-term treatment outcomes are dependent on healthy systemic functioning, but the family impact of a treatment is rarely evaluated, so IBM Watson services are used for combination these children [50]. It is one of IBM's software products that have several services that are used to provide interaction dialog. The Watson conversation service is used to implement the interaction dialog, Text-to-Speech, and Speech-to-Text services to enable the voice interaction [51]. Watson assistant solutions have the most impact that are built for proactive assistants with when they are designed to be personal and portable. IBM's assistant is essentially different than that of traditional web applications or mobile especially when the assistant has a combination of text and voice or a voice interface [52].

## 4. The Proposed System

The flowchart of the proposed system including hardware and software implementation is illustrated in Figure 3.

### 4.1. Hardware Implementation

As mentioned previously, autistic children face a problem in expressing their emotions and in communicating with others. So, emotion refers to a feeling that can be caused by the situation the person is in. In this system, some vital parameter like heart rate is measured. The proposed system takes the heartbeat as input, while the output will be one of four suitable emotions such as, sad, happy, excited, and angry. As shown in Figure 4 the system architecture is split into two main modules, hardware and software. The hardware prototype can be performed by the following steps:

1. The heartbeat sensor is attached to the ASD child to provide the data in a numeric form.
2. The signal pin of the pulse sensor is connected to an analog pin of ESP32, where the board must be connected to a Wi-Fi network.
3. The ESP32 sends the data to the Firebase (web service) for classification.
4. Call SVM algorithm to determine the state.
5. Convert the state of the child to emotion using the mobile application.
6. Monitor real-time emotions that can be viewed remotely via a mobile phone.

### 4.2. Software Implementation

Now, we introduce the description of elements used in software implementation such as android, computer graphics, and 3D modeling. Android is an operating system of the mobile based on open-source software, which is designed primarily for touchscreen mobile devices like smartphones and tablets. Computer graphics is the visual image or design displayed on a variety of surfaces, including a computer monitor, a canvas, a wall, or a sign for entertainment and providing information. The process of creating any object and surface as a representation by handling polygons, edges, and vertices in simulated 3D space is known as 3D modeling [53–55].

The heartbeat sensor is used to read the heart rate of the child and convert it to some states. Then, this state is converted to emotion using an mobile program as reported in Figure 5 which help us know the state of the autistic child. After that, the graphical design is used to help this child adapt to anyone who cannot contact. Also, we have scheduling tasks in this application that help the parents remember the child's activities. The web services platform gives the flexibility to manage and store data. For more explanation, the software can be performed using the following steps:

1. Use a web service that includes the SVM algorithm to classify numeric values into a suitable state using Python Language.
2. Create a mobile application using Android studio software.
3. Connect this application via the Internet with the web service Firebase.
4. Build the 3D graphic model using IBM Watson Assistant.
5. Masking the image in the 3D model, which communicates with the guardian.

In the system, data will be classified depending on ranges of heart rate, and the model will be retrained and tested by percent 70 : 30. Finally, send the appropriate state of the child, whether happy, sad, excited, or angry to the mobile of the guardian. In the mobile part, there are some pages that contain the components of the application including login page to sign in into the application, registration page to sign up into the application for the first time, notification page to send emotions as a notification with child state, and suggestions to help the guardian treat the child in any of the cases coming from the sensor, and the scheduling page concerns the child, which includes the times of treatment and appointments of doctors that help the mother know the exact time of treatment of the child. The IoT is increasingly allowing the integration of devices capable of connecting to the Internet and providing information in real-time to the parents via autism care application. This application can assist parents in understanding their autistic children from the emotion displayed on the mobile and help them communicate with others easily.

## 5. Experimental Results and Discussion

In this section, we experimentally evaluate the efficiency of the proposed autism care system using data determined from the center of autistic children at young ages between 4 and 12 years. These data depend on the heart rate for these children based on Homocysteine. All experiments are performed on a Core I7 windows10 machine with a 16 GB memory, and Python language and IBM Watson assistant for unity are installed for producing the 3D graphic image.

### 5.1. Preprocessing Steps

The preprocessing steps have been explored before testing stage to achieve efficient results from the system software. In the first step, filter-based feature selection methods use statistical measures to score the correlation between input variables that can be filtered to choose the most relevant features. As shown in Figure 6, the heart rate measurement before and after applying filter selection method is according to different number of features. Therefore, this will lead to improving the prediction performance of the model and accurate heart rate measurement while reducing the number of features.

In the second step, classification scheme provides machine learning step according to support vector machine. Through SVM, we obtain evaluation matrix known as accuracy, which can be used as a measurement of the heart rate. As illustrated in Figure 7, the relationship between heart rate and classification accuracy is achieved using SVM technique. As the heart rate ranges from 70 to 100 bpm, the accuracy percentage ranges from 98 to approximately 99,8. Thus, a high number of features can lead to lower classification accuracy and vice versa.

### 5.2. Sample Test Scenario

We test the system software according to many criteria including, unity, integration, validation, alpha, and beta testing. In unity testing, every component of our proposed system is tested separately such as heartbeat sensor, machine learning model, mobile application, and graphic model. In integration testing, two or more of these components are combined for testing them separately. In the validation test, it should be ensured that if the tested and developed application satisfies its functionality requirements, the business requirement logic or scenarios have to be tested in detail. So, all the critical functionalities of an application must be tested here. Moreover, alpha testing is performed to distinguish bugs before publishing the product to real users or the public. It is exploited by in-house software engineers. It is the final testing stage before the software is released into the real world. Finally, we have beta testing in which developers are used for testing a sample version of the software to be available for downloading from the web [56]. In the software, we have four possible scenarios for testing as follows:

Test scenario 1: testing the heart rate values to classify it to a suitable state.
     Input: numeric values.
     Output: state.
Test scenario 2: testing the connection between ESP32 and the web service by checking if Wi-Fi sending the state or not.
     Input: ESP32 with WiFi connection.
     Output: data stored in Firebase.
Test scenario 3: testing the login and authentication functionality.
     Input: username and password.
     Output: accept or reject.
Test scenario 4: testing if the graphical image is displayed parallel with the voice or not.
     Input: 3D graphic image.
     Output: voice merged with 3D model.

The mobile application has pages that contain some contents as follows:

(1) Login page: this page has the username and password. Also, it has a button for the registration page if the user is not registered.
(2) Registration page: a page that enables the user to register his data to be able to use the application. After the user logs in, the user sees a new page containing three contents:
  1. Emotion page: a page which has the child's feelings from the sensor with suggestions to help the guardian act with the child in case of situations coming from the sensor.
  2. Graphic page: it has a picture of virtual people from the real world, which are transformed into three-dimensional graphics to help the child adapt to the outside community.
  3. Scheduling page: this is for the guardian to include the child's activities through a day by setting tasks and time for each.

### 5.3. Heart Rate Measurement

Heart rate usually speeds up slightly as a child inhales and slows as he exhales known as respiratory sinus arrhythmia (RSA). RSA serves as a surrogate for the activity of the nervous system, which regulates heart rate and breathing, among other functions. The fluctuations are responsible for regulating emotions and attending to social cues. As listed in Table 1, the proposed system was tested on 20 children with two recordings per child. The first recording is conducted on the age of the child in which a resting supine is provided a baseline measurement of the resting heart rate (70 bpm). The second was taken after a change in the child mode, which captured elevated cardiac activity. Different emotions through the autonomic nervous system affect heart rate, and this difference in the heartbeat is obvious when the child's mood changes.

### 5.4. Emotion Analysis

In Figure 8, we illustrate that the change of heart rate for 30 autistic children in the testing dataset leads to the change in their emotions (angry, happy, excited, and sad) using the proposed system. The specific heart rate patterns were investigated to cooccur with challenging behaviors in children diagnosed with ASD. Abnormal heart rate responses to stressors were also noted, and we compared the level of homocysteine and other biomarkers in children with autism to corresponding values in age-matched healthy children. It is clear that the child can be angry when his heart rate is between 80 and 180 bpm, while in the case of happiness the heart rate is between 60 and 100 bpm. Moreover, when it ranges between 110 and 140 bpm, the child is feeling excited. Finally, the child is being sad when his heart rate is between 160 and 185. Thus, the pulse can be a strong indicator for detecting emotions, especially in autistic children. Likewise, parents can easily interact with their autistic children efficiently using our technology.

### 5.5. Performance of Classification

Depending on the extracted features from the datasets, the classification models should be tested by trying a combination of various machine learning algorithms such as Random Forest (RF), KNN, and SVM to determine the appropriate one for the classification of data set. As reported in Table 2, we found that RF and KNN have the accuracy percentage with 95 and 97, respectively. The accuracy is enhanced using ensemble techniques with SVM that achieves an accuracy of 99.8. So, the SVM is the best algorithm that can be used for classifying the data set to achieve our goal of emotion analysis for the ASD children in accurate and effective using the heart rate.

## 6. Conclusions

In this paper, we proposed an intelligent system with AI-enabled Internet of Things to help the autistic child adapt to the surrounding environment by determining the emotional state of the child through a sensor that reads the child's heartbeat that is classified by the machine learning models. Four classification models are tested, where SVM and RF were the best for this task. Then, a notification is sent with the child's state to the guardian with recommendations suitable for the child's emotion. Further, the application interface of the proposed system allows the guardian to remember a child's activities. In addition, this application helps autistic children who suffer from an eye contact problem, through interacting with the 3D graphical model. The proposed system attempts to obtain emotional feelings in a group of autistic children by analyzing heart rate before, during, and after challenging behaviors. To achieve more security for the data, cloud computing services can be used to improve the results to be more accurate. Moreover, optimization algorithms can be performed to help parents in improving the behavior of their Autistic children in an easy way using this technology.

## Figures and Tables

**Figure 1:** Hardware components used for building the proposed system.

**Figure 2:** Linear separation of SVM.

**Figure 3:** Flowchart of the proposed system.

**Figure 4:** The general architecture of the proposed system.

**Figure 5:** GUI of the proposed mobile application for the proposed system.

**Figure 6:** Heart rate before and after filter selection based on number of features.

**Figure 7:** Relationship between heart rate and classification accuracy achieved by SVM technique.

**Figure 8:** Relationship between emotions and mean heart rate among 30 autistic children.

**Table 1:** Child's emotion according to change in heart rate.

Emotion	Average heart rate (bpm)
Angry	80
Angry	150
Angry	165
Happy	60
Happy	70
Happy	75
Happy	85
Happy	90
Happy	100
Excited	110
Excited	120
Excited	130
Excited	140
Sad	160
Sad	160
Sad	165
Sad	170
Sad	175
Sad	180
Sad	185

**Table 2:** Comparison between four machine learning classifiers.

Algorithm	KNN	RF	SVM
Accuracy %	95	97	**99.8**
Precision %	81	83	**88**
Best	95	97	**99.8**
Worst	90	93	**95.8**

## Data Availability

No data were used to support this study.
